The article "Spine Medical Image Segmentation Based on Deep Learning" was retracted in 2023. Reasons: signs of a paper mill; suspected computer-generated content; unreliable results or conclusions; concerns about the data.

# Spine Medical Image Segmentation Based on Deep Learning

**DOI:** 10.1155/2021/1917946

**Published:** 2021-12-15

**Authors:** Qingfeng Zhang, Yun Du, Zhiqiang Wei, Hengping Liu, Xiaoxia Yang, Dongfang Zhao

**Affiliations:** ^1^Beijing University of Chinese Medicine Third Affiliated Hospital/Spin,Department, Beijing 100029, China; ^2^The Second School of Clinical Medicine, Beijing University of Chinese Medicine, Beijing 100078, China; ^3^Dongfang Hospital Beijing University of Chinese Medicine/Orthopaedics, Beijing 100078, China

## Abstract

The aim was to further explore the clinical value of deep learning algorithm in the field of spinal medical image segmentation, and this study designed an improved U-shaped network (BN-U-Net) algorithm and applied it to the spinal MRI medical image segmentation of 22 research objects. The application value of this algorithm in MRI image processing was comprehensively evaluated by accuracy (Acc), sensitivity (Sen), specificity (Spe), and area under curve (AUC). The results show that the image processing time of fully convolutional network (FCN) algorithm and U-Net algorithm is greater than 6 min, while the processing time of BN-U-Net algorithm is only 5–10 s, and the processing time is significantly shortened (*P* < 0.05). The Acc, Sen, and Spe results of BN-U-Net segmentation algorithm were 94.54 ± 3.56%, 88.76 ± 2.67%, and 86.27 ± 6.23%, respectively, which were significantly improved compared with FCN algorithm and U-Net algorithm (*P* < 0.05). In summary, the improved U-Net network algorithm used in this study significantly improves the quality of spinal MRI images by automatic segmentation of MRI images, which is worthy of further promotion in the field of spinal medical image segmentation.

## 1. Introduction

The spine plays a key role in the normal activity and regulation of the central nervous system in which all parts of the human body are the spinal cord. The slight injury to the spine in daily life may cause the patient's whole body to suffer injury. At the same time, there are a large number of neurons in the spine, which makes the human body suffer unbearable pain [1, 2]. The spine is one of the most important parts of the human body. Medical imaging of the spine can be performed at different ages. With the continuous progress of society and the increasing pressure of human work and life, sedentary work or long-time study are gradually leading to the abnormality of human spine [3]. Spinal diseases often occur in all kinds of people and ages. Back pain affects the normal work and study of individuals, has become a worldwide health problem, and has attracted the attention of a large number of clinical experts [4]. After research, the pain caused by spinal injury can be treated by physical and biochemical techniques.

At present, MRI technology is one of the most commonly used imaging technologies in clinical spine examination [5]. Compared with X-ray, CT, and other equipment, MRI imaging examination not only has no ionizing radiation but also has the comparative resolution ability of soft tissue that other equipment cannot compare [5]. For spinal lesions, MRI can detect changes such as intervertebral disc degeneration, protrusion, or bulging at an early stage. MRI can observe multiple vertebral bodies and intervertebral discs at a time, which avoids the limitation that other imaging devices can only selectively perform several intervertebral disc imaging [6, 7]. However, there are problems such as blurred edges of spinal MRI images, low discrimination with the surrounding areas, inability to show good tissue morphology, and chaotic structural imaging, which make the application of image segmentation technology in spinal MRI imaging more and more [8]. Deep learning is a kind of machine learning algorithm, which can achieve supervised, semisupervised, or unsupervised image processing by using multiple layers to gradually extract higher-level features from the original input [9]. Convolutional neural network (CNN), as a feedforward neural network, is one of the most widely used. Its artificial neurons can respond to a part of the surrounding units within the coverage to achieve efficient processing of large images [10]. In recent years, deep learning technology has been widely used in the segmentation of various medical images. Various deep learning algorithms emerge endlessly, which make the quality of medical images significantly improved. For example, the semiautomatic segmentation of spinal MRI images is realized by deep learning algorithm to improve the edge blur and type matching limitation of conventional MRI images. In view of the obvious difference between the gray levels of intervertebral disc and vertebra in MRI images, the noninitial state set model is added to the spinal medical image, so as to realize the effective segmentation of intervertebral disc MRI images [11].

Based on this, in order to further improve the segmentation quality and accuracy of spinal image, this research studies and proposes an improved U-Net image segmentation method. By constructing the network model, this research explores the MRI image features and effects processed by deepening the U-Net network image segmentation algorithm, to provide more reference for doctors in clinical practice.

## 2. Method

### 2.1. Full Convolution Neural Network

Since the advent of the convolutional neural network (CNN), it has been widely used in medical image classification, target recognition, and semantic segmentation, which has made great achievements in the field of medical imaging. However, the single use of CNN technology for medical image segmentation is not ideal. The segmentation technology has extremely high requirements for pixels, and different images will be used as detection objects, so it puts forward great requirements for the segmentation technology. To solve the abovementioned problems, Zhu et al. [12] applied the full convolutional network (FCN) to medical image segmentation. The full convolution neural network samples the output of the network with a smaller size to a larger size by converting the convolution layer and using the sampling layer, which makes it possible to obtain a wider receptive field by using the full convolution neural network, which can input images of various sizes for different levels of segmentation at the same time. The structure of the full convolution neural network is shown in Figure 1. The network combines the deep feature map with rough spatial location information but rich semantic information with the shallow feature map with poor semantic information but fine spatial location information, so as to further improve the segmentation results of the network.

### 2.2. Improved U-Net Network

In recent years, the emergence of U-Net network has solved a large number of image segmentation problems that cannot be overcome by previous technologies. The full convolution neural network generally processes the input image by downsampling and directly upsampling to the original image size. Unlike the full convolution neural network, U-Net divides different network frameworks by constructing encoders [13]. In this study, it tries to add a specification layer (BN layer) between different convolution layers and activation layers and at the connection between each inner layer and activation layer, so as to improve the U-Net network. It believes that the data of a certain layer in the convolution network are normalized in batch, and *R*_*xy*_^*a*^ refers to the output of *X* neurons in layer *y* when the model is trained to the *a*-th data. *F*_*xy*_ refers to the average output of the *x*-th neuron in layer *y*, and *K*_*xy*_ represents the standard deviation of the output of the *x*-th neuron in layer *y*. The output value *P* obtained after batch normalization is as follows:

(1) $$\begin{array}{c} P=\frac{R_{xy}^{a}-F_{xy}}{K_{xy}}. \end{array}$$

The mean value of neuron output is

(2) $$\begin{array}{c} F_{xy}=\frac{1}{t}\sum_{a=1}^{t}R_{xy}^{a}. \end{array}$$

The standard deviation of neuron output is

(3) $$\begin{array}{c} K_{xy}=\sqrt{b+\frac{1}{t}\sum_{a=1}^{t}{\left(R_{xy}^{a}-F_{xy}\right)}^{2}}. \end{array}$$

The values of *b* and *t* are constant. The output of batch normalization using the specification layer activation function is as follows: input *n* adds the weight through the weight *L* and finally obtains the output through the activation function to obtain the following equation:

(4) $$\begin{array}{c} U=f\left(BN\left(\sum_{a=1}^{t}L_{x}N_{x}\right)\right). \end{array}$$

### 2.3. Image Segmentation Algorithm Based on Improved U-Net Network

In this study, the BN-U-Net network is constructed to segment the spinal MRI image, the connection mode is redesigned to aggregate the scale features of different decoding subnetworks, and a flexible feature aggregation method is formed through pruning to improve the learning and reasoning speed and greatly improve the segmentation accuracy. Spine medical image segmentation is simple and easy to understand. Among the results presented, the first column of the original spine image is input. After the original image is input into the segmentation environment, the second column of the image is the result obtained by identifying the model and selecting the segmentation target area. In order to ensure the segmentation accuracy and facilitate the judgment of pixel division, it marks the segmentation target, selects the regional background target in the red mark box, and obtains the third column of segmentation results through algorithm segmentation, as shown in Figure 2.

Figure 3 is the flow chart of spine segmentation optimization. The optimization framework includes two organizational structures. First, the spine image will generate a structural image with the same size as the original image after the network segmentation; then, the obtained structure segmentation graph is processed by the undirected graph to reconstruct and organize the energy function. After the abovementioned two steps, a perfect and clear high-quality segmentation image is obtained.

## 3. Experiment

### 3.1. Experimental Data

The data of this study come from the public dataset annotated T2 commonly used in spine segmentation-related algorithms weighted MR images of the lower spine (MR lower spine). This dataset is given by Hofmann et al. [14]. This dataset contains sample images of 22 people and corresponding manually segmented real images. After transverse slicing, the images without spine are removed, and the dataset is appropriately expanded through geometric transformation.

### 3.2. Evaluating Indicator

In order to measure the advantages and disadvantages of the algorithm, the evaluation indexes such as accuracy, sensitivity, specificity. and area under the curve (AUC) are used. In this study, the predicted and actual MRI image segmentation results are evaluated as true, which is defined as a; if the forecast is false and the actual is true, it is defined as b; if the forecast is true and the actual is false, it is defined as c; and the forecast is false and the actual is false, which is defined as d.  Table 1 shows the specific relationship.

The accuracy of the measured samples (as shown in equation (5)) is the proportion of the total number of MRI samples; sensitivity, also known as recall rate, represents the proportion of correct samples determined by MRI images in all correct samples actually released, as shown in equation (6); specificity refers to the proportion of targeted release error samples judged by MRI in all actual targeted release error samples, as shown in equation (7); and the area under the curve (AUC) refers to the area of the part surrounded by the curve and the coordinate axis. This value will not be greater than 1, as shown in equation (8).

(5) $$\begin{array}{c} \text{Accuracy}=\frac{a+d}{a+b+c+d}\times 100\%, \end{array}$$

(6) $$\begin{array}{c} \text{Sensitivity}=\frac{a}{a+c}\times 100\text{\%,} \end{array}$$

(7) $$\begin{array}{c} \text{Specificity}=\frac{a}{a+b}\times 100\text{\%,} \end{array}$$

(8) $$\begin{array}{c} \text{AUC}=\frac{d}{c+d}\times 100\%. \end{array}$$

### 3.3. Statistical Analysis

SPSS 24.0 software was used for statistical analysis, which was expressed as mean ± standard deviation ($\overset{¯}{x}$ ± *s*). The comparison between groups was carried out through one-way ANOVA. When the homogeneity of variance was met, the least significant difference (LSD) method was used to test, and when the variance was uneven, the T2 test was used to test the level *α* = 0.05, *P* < 0.05.

## 4. Discussion

### 4.1. Network Output Spinal MRI Images

In this study, the spinal MRI image segmented by the constructed algorithm is transformed into gray image, and the probability that different pixels belong to various categories in the represented image is highlighted according to the depth of image gray.  Figure 4 is the probability prediction gray map of spine image output by the network. It can be seen from the figure that the gray level of the edge and surrounding of the probability prediction map is slightly lighter than that of other parts, which indicates that the pixels in this part are likely to belong to the spine, the gray level of the surrounding background is slightly deeper than that of this part, and the background part may be on spine. In addition, it also shows that the spinal MRI image segmented by this algorithm can clearly distinguish the spinal and nonspinal parts, and the automatic segmentation algorithm constructed in this study is very close to the real segmented image and has high similarity.

### 4.2. Segmentation Results of Spinal MRI Images Based on Deep Learning Algorithm

Three groups of representative spinal MRI images are randomly selected from the dataset used in the study, and these images are input into the network model constructed in this study for segmentation. The segmentation results are shown in Figure 5. The spinal MRI image segmentation obtained by U-Net algorithm is generally similar to that obtained by BN-U-Net algorithm, but compared with U-Net algorithm, the spine MRI image segmentation of BN-U-Net algorithm has significantly improved the image definition, refined the segmentation of spine edge image, and can more accurately identify the related lesions of the spine.

### 4.3. Comparison of Image Segmentation Results of Different Algorithms

The accuracy, sensitivity, specificity, and imaging time of segmented images with different algorithms are counted, and the data statistics table (Table 2) is obtained. The results show that the accuracy, sensitivity, and specificity of BN-U-Net segmentation algorithm are 94.54 ± 3.56%, 88.76 ± 2.67%, and 86.27 ± 6.23%, respectively. Compared with FCN algorithm and U-Net algorithm, the accuracy, sensitivity, and specificity of BN-U-Net segmentation algorithm have been significantly improved, and the difference is statistically significant (*P* < 0.05). In addition, the image processing time of FCN algorithm and U-Net algorithm is 60–360 s and 180–300 s, respectively, while that of BN-U-Net algorithm is only 5–10 s, which is significantly shortened (*P* < 0.05). This shows that compared with FCN and U-Net algorithms, the BN-U-Net image segmentation algorithm designed in this study can significantly improve the segmentation accuracy, sensitivity, and specificity of spinal MRI images, so as to further improve the MRI image diagnosis accuracy of spinal related diseases. The image segmentation time is greatly shortened, and the MRI image processing efficiency is significantly improved. It can further meet the needs of clinical diagnosis of spine-related diseases. However, the accuracy of the algorithm is not improved enough, and the details of image segmentation are rough.

## 5. Conclusions

In this study, an improved U-Net network automatic segmentation algorithm was designed and applied to the segmentation of spinal MRI medical images of 22 research objects. The results show that the improved U-Net network automatic segmentation algorithm greatly shortens the MRI image processing time compared with the FCN algorithm and the U-Net algorithm, and the accuracy, sensitivity, and specificity of image segmentation are significantly improved. Therefore, the BN-U-Net segmentation algorithm can further improve the segmentation quality and accuracy of MRI images of the spine and has an active role in the characteristics and processing effects of MRI images. However, there are still some shortcomings in this study; for example, the sample size of patients with spinal MRI images included in the study is small and the source is single. In addition, the improved U-Net network automatic segmentation algorithm is slightly insufficient in terms of imaging clarity. Future research hopes to further optimize the algorithm to improve this problem. In conclusion, the improved automatic segmentation algorithm based on U-Net network can significantly improve the automatic segmentation efficiency of spinal MRI images and improve the clinical diagnosis accuracy of spinal diseases, which is worthy of further promotion. Moreover, the method proposed in this study can not only solve the segmentation problem of spinal image well but also provide more processing approaches for other types of medical images.

## Figures and Tables

**Figure 1:** Full convolutional network.

**Figure 2:** Spinal MRI image segmentation.

**Figure 3:** Spine segmentation optimization framework.

**Figure 4:** Probabilistic prediction gray image of spine image output from the network. (a) The input image, (b) the real segmented image, and (c) the probability prediction diagram.

**Figure 5:** Segmentation results of spinal MRI images. The first line is the original image input. *X* represents U-Net algorithm segmentation graph. *Y* represents the BN-U-Net algorithm segmentation graph. 1, 2, and 3 represent spinal MRI images of different patients.

**Table 1:** Confusion matrix.

	The prediction is true	The forecast is false
Actually true	a	b
Actually false	c	d

**Table 2:** Comparison of spinal MRI image segmentation results based on different algorithms.

Algorithm	Accuracy (%)	Sensitivity (%)	Specificity (%)	Time (s)
FCN	89.27 ± 3.68	82.56 ± 2.33	77.43 ± 6.54	60–360
U-Net	90.35 ± 2.14	84.48 ± 1.98	77.92 ± 6.79	180–300
BN-U-Net	94.54 ± 3.56^*∗*^	84.76 ± 2.67^*∗*^	86.27 ± 6.23^*∗*^	5–10^*∗*^

^*∗*^Significant difference in analysis of variance (*P* < 0.05).

## Data Availability

The data underlying the results presented in the study are available within the manuscript.
